# Analysis of body heat tolerance of workers in a simulated warm environment based on linear mixed model

**DOI:** 10.1371/journal.pone.0279170

**Published:** 2022-12-22

**Authors:** Mohsen Aliabadi, Masoud Shafiee Motlagh, Rostam Golmohammadi, Rashid Heidarimoghadam, Maryam Farhadian

**Affiliations:** 1 Center of Excellence for Occupational Health, Occupational Health and Safety Research Center, Hamadan University of Medical Sciences, Hamadan, Iran; 2 Center of Excellence for Occupational Health, Research Center for Health Sciences, Hamadan University of Medical Sciences, Hamadan, Iran; 3 Department of Ergonomics, Research Center for Health Sciences, Hamadan University of Medical Sciences, Hamadan, Iran; 4 Department of Biostatistics, Researches Center for Health Sciences, School of Public Health, Hamadan University of Medical Sciences, Hamadan, Iran; US Army Research Institute of Environmental Medicine, UNITED STATES

## Abstract

Workers’ heat tolerance plays a crucial role in maintaining their health and performance in hot environments. This study aimed to empirically analyze the body heat tolerance of workers under a simulated warm environment. Twenty healthy male workers from the typical light metal industry (age: 23.15±2.45 years) were participated in the experimental study. Workers were exposed to two thermal environments (Ta = 22°C, RH = 35%, and Ta = 35°C, RH = 35%) in a simulated moderate workload in a climate-controlled room. The maximal aerobic capacity (VO_2_ max) and body fat mass of workers were determined. The heat tolerance indicators were determined based on heart rate (HR) and ear temperature (ET) before and after each experiment. A linear mixed model was employed to analyze body heat tolerance indicators using the SPSS statistical package. All physiological responses significantly increased in the warm air condition compared to the thermoneutral condition. The HR and ET increased by an average of 14 bpm and 0.75°C, respectively (p<0.05). The mixed model could accurately predict heat tolerance indicators (r = 0.95 and r = 0.97) so that the VO_2_ max and body fat mass were identified as the main individual influential factors. The VO_2_ max showed significant correlation with urinary specific gravity (r = -0.55, p<0.05), HR (r = -0.59, p<0.05), and ET (r = -0.57, p<0.05) in warm environment. The model confirmed that physical fitness is critical in increasing heat tolerance in warm environments. It can be a helpful screening tool for properly selecting workers in occupational medical examinations for working in warm air conditions. It is proposed that workers’ regular exercise and lifestyle modifications can strengthen their heat tolerance.

## 1 Introduction

Exposure to warm air conditions in the workplace can directly or indirectly affect employees’ physiological responses, such as body temperature, metabolism rate, heart rate (HR), and blood pressure [1–3]. It can cause heat-related illnesses, including heat exhaustion, muscle cramps, heatstroke, heat rashes, and neuropsychiatric disorders [3–5]. Reduced work performance caused by heat stress also increased the rate of human errors and accidents in the workplace [3, 6–10]. Moreover, the most dangerous consequence of overexposure to heat in the workplace is heatstroke, leading to death in more severe cases [3, 11].

The main factors are effective in causing heat strain, including essential environmental factors, such as ambient air temperature, radiant air temperature, air velocity, relative humidity (RH), and underlying personal characteristics, such as age, weight, acclimatization level, metabolism rate, and health status [3, 12–14]. In addition to the aforementioned environmental and underlying factors, some secondary body physical factors may affect the level of body heat tolerance. The most critical factors include body fat mass, body volume to surface ratio, physical fitness, and maximal aerobic capacity (a cardiopulmonary index of maximal oxygen uptake) [1, 3, 15, 16]. Maximal aerobic capacity (also known as VO_2_ max or peak oxygen uptake) indicates the maximum rate of oxygen transport to the muscles. It depends on cardiac output and oxygen used by the muscles [17, 18]. The maximal aerobic capacity is frequently used to measure the fitness of the cardiorespiratory system [3, 15, 19, 20].

Some researchers practiced the protocol for the determination of body heat tolerance. Moran et al. showed the applicability of the heat tolerance test (HTT) as a relatively accurate screening tool in identifying individuals’ tolerance/intolerance to heat [21]. HTT has defined human exposure to thermal air conditions in a climatic chamber while walking on a treadmill dressed in light cloth. This way, the heat strain indicators such as body temperature and heart rate are continuously monitored [21]. The experiment study on thermal comfort and body heat tolerance is frequently employed to investigate cognitive and physiological responses to different thermal conditions in diverse populations [22–24]. Lu et al. studied different people’s body’s physiological responses to heat in three climate conditions: warm-dry, warm-humid, and mild air temperatures. They found that VO_2_ max and weight significantly affect the body’s physiological response to subjects’ exposure to heat [16]. Havenith et al. showed that individual characteristics play a significant role in determining the responses of body core temperature in all studied environments [25]. Lisman et al. studied the relationship between heat intolerance and body anthropometric dimensions and fitness. They indicated that VO_2_ max was the most influential factor in heart rate and core body temperature during the heat tolerance test [26]. Mee et al. found that some variables of body mass index, HR, VO_2_ max, rectal temperature, and ST can be considered the most influential variables in the heat tolerance level [27]. Some studies have demonstrated that individuals with a lower VO_2_ max have a reduced ability to thermoregulate relative to individuals with a higher VO_2_ max during exercise scenarios [28, 29].

It seems that prediction models for analyzing the body responses in any climatic conditions are most helpful in implementing effective preventive measures. Statistical modeling provides one of the best solutions to tackle these complex phenomena. Linear mixed models (LMMs) are increasingly used for data analysis in various physical, biological, and social disciplines [30–35]. However, few studies reported using these statistical approaches to predict thermal strain [32, 33, 35].

Moreover, most of the aforementioned studies about the analysis of heat tolerance were conducted on athletes and the military population, whose individual characteristics and nature of activities are different from the working environment. There is a dearth of studies on the effects of these underlying factors on the thermal comfort of workers in warm working environments. An essential measure in preventing heat strain in warm workplaces is the proper selection of workers in medical examinations [36]. In this regard, explaining the role and effects of the different influential risk factors on body heat tolerance can facilitate selecting workers appropriate to working climate conditions. This study aimed to empirically analyze the body heat tolerance of workers under a warm environment based on a linear mixed model.

## 2 Materials and methods

### 2.1 Participants

Twenty healthy male workers from the typical light metal industries of Hamadan city (located in the west of Iran) were selected. The workers with a history of smoking, diabetes, hypertension, hyperthyroidism, cardiovascular disease, kidney disease, sleep disorders, and heat-related illnesses were excluded from the study. They were recommended not to use caffeine or other stimulants 12 hours before the experiments. This study was approved by the Ethics Committee of Hamadan University of Medical Sciences (ethic code: IR.UMSHA.REC.1394.439). All methods were performed according to the guidelines and regulations approved by the Hamadan University of Medical Sciences Ethics Committee. After being informed about this research, written consent was obtained from the participants, which the ethics committee approved. They were also informed of the aim and method of the study. If the body temperature reaches more than 38.5 degrees Celsius, the person feels dizzy, nauseous, or weak, or the heart rate reaches the maximum threshold according to Eq (1), the experiments will be stopped [3, 37].


$${HR}_{max}=180-age$$ (1)

Where HR_max_ is the maximum threshold of heart rate (bpm), age is the person’s age (years)

### 2.2 Experiment setup

The experiment was carried out using a within-participants design, where all participants were tested under two experimental environments, thus acting as their own controls. The flowchart of different steps of the experiments is presented in Fig 1.

**Fig 1:** The flowchart of different steps of the experiments.

The experimental environment was a climate-controlled room with dimensions of L×W×H = 3.70×2.40×2.70m. It was possible to set and fix the chamber’s thermal environments using an air-conditioner system within -10 to 50°C and relative humidity of at least up to 90%. It is equipped with an automatic air oxygen regulation system. The room has two LED lamps which provide a luminance of 300 lux. Fig 2 displays the climate-controlled room. During the experiment, the thermometer sensors installed on the room’s wall continuously monitored the thermal environments, including air temperature and relative humidity.

**Fig 2:** Climate-controlled room for experiments.

The participants were exposed to two conditions of thermal environments simulated in the climate-controlled room: thermoneutral (Ta = 22°C, RH = 30%) and warm (Ta = 35°C, RH = 35%). In both environments inside the climate-controlled room, a treadmill (Elite T5, Horizon) was used to simulate a moderate workload (130–200 w/m^2^) with a treadmill speed of 3.5 km/h with a slope of 2% [38]. The participants were walked on a treadmill for 30 minutes in each environment. Furthermore, the clothes thermal insulation of the participants was maintained at 0.75 clo by the recommended ISO 9920:2007 standard [39].

### 2.3 Maximal oxygen uptake (VO_2_ max)

The step test was used to determine the maximal oxygen uptake (VO_2_ max) of participants according to the standards proposed by the American College of Sports Medicine (ACSM) [40]. For this purpose, the subject had to go up and down 40 cm-high stairs in 3 minutes; then, the frequency of going up and down the stairs per minute was obtained. Subsequently, VO_2_ max was calculated and expressed in units of liters (l) of O2 per minute (min) using participants’ weights in kilograms and HR measured immediately after the test based on Eq (2).


$$VO_{2\max}=\frac{AG(131.5\times VO_{2})}{HR+GF-72}$$ (2)

Where VO_2_ max is the maximal oxygen uptake (l/min), VO_2_ is the oxygen consumption at a steady-state (l/min), HR is the heart rate (bpm), GF is the sex factor (for men ten and women zero), AG is the age correction factor that was calculated by Eq (3),

AG=1.12−0.0073age (3)

Where age is the person’s age (years),

$$VO_{2}=(0.35\times f)+(2.395\times f\times h)$$ (4)

Where f is the frequency of going up and down the steps (step per minute), h is the step height (m), and VO2 is the oxygen consumption at a steady-state (ml/kg/min).

### 2.4 Body composition analysis

Body fat and muscle masses were measured using a body composition analyzer (N20, AIIA Communications Inc). Moreover, the hydration status of the participants must be the same for two experiment sessions. In this way, the participants’ urine specific gravity (USG) was measured and recorded in each experiment scenario using a digital refractometer (PAL-10S, Atago, Japan). The experiment session was cancelled if the subject’s hydration level was unusual. USG is widely accepted as a convenient and reliable indicator of hydration status [3, 41–44].

### 2.5 Body heat tolerance indicators

According to the recommended ISO 9886:2004 standard [43], participants’ physiological responses, including heart rate (HR), ear temperature (ET), and skin temperature (ST), were measured before and after walking on a treadmill to determine their heat tolerance. The subjects’ ET was measured with an ear thermometer (TH839S; OMRON Instruments). The main reason for selecting ET to represent body temperature was the simple measurement of ET using an accurate and non-invasive thermometer [45]. It should be noted that the invasive measurement of body temperature indicators, such as the rectal temperature, can lead to participants leaving the study.

For measuring ST (forehead temperature), an infrared thermometer (TG165; FLIR Instruments) was used. The subjects’ heart rate was measured using a monitor device (E600; POLAR Instruments). This device had a sensor mounted on the chest and a display placed on a wrist strap. The sensor communicated with the display via Bluetooth and showed the heart rate. All physiological responses were measured three times in each step, and their mean was recorded for each measurement. It is noteworthy that before the commencement of the treadmill test, participants sat quietly on a chair for 15 minutes and drank 250cc of water at room air temperature to keep the standard baseline heart rate.

### 2.6 Statistical analysis

Data normality was tested using the Kolmogorov-Smirnov test. When data were normally distributed, they were analyzed using the paired-sample and student T-tests. The significant relation among some features was analyzed using Pearson correlation. Wilcoxon’s tests will consider when the data distribution is not normal. The significant level for all tests was set at 5%. The linear mixed model (LMM) was also run to evaluate different influential risk factors on heat tolerance indicators such as heart rate and ear temperature. LMM describes the relationship between a response variable and other explanatory variables that have been obtained along with the response [30, 31]. In these analyses, the participant was added to the model as a random variable for grouping the data for each participant to show that the same participant was measured several times. This means that the intercept is a random variable rather than a constant one, i.e., the intercept varies between the participants [34]. Data were analyzed in SPSS software (ver.22, Chicago, IL, USA).

## 3 Results

The results of the demographic and body characteristics of the participants are presented in Table 1. The results showed that the mean BMI of the participants is approximately in the normal range.

**Table 1:** Demographic and body characteristics of the participants (n = 20).

Variable	Mean ± SD	Min	Max
Age (yrs)	23.15**±**2.45	20.00	26.00
Height (m)	1.77**±**0.05	1.69	1.89
Weight (kg)	70.75**±**11.99	48.00	98.40
Body mass index (kg/m^2^)	22.39**±**3.20	16.4	28.38
Muscle mass (kg)	53.40**±**7.10	44.50	71.30
Body fat mass (kg)	13.80**±**6.10	2.00	24.00
Vo_2_ max (lit/min)	2.13**±**0.40	1.40	2.82

### 3.1 Results of the heat tolerance indicators

Table 2 presented the body’s physiological responses before and after walking on a treadmill in thermoneutral and warm conditions. It can be seen that, in the warm air condition, the mean HR, ET, and ST were significantly higher than in the thermoneutral condition (p<0.05). There was no significant difference between the baseline HR before walking on a treadmill in thermoneutral and warm conditions (p = 0.154). Based on the guidelines for interpreting urine-specific gravity readings, the participants have marginally adequate hydration in two air conditions (USG = 1.02±0.01).

**Table 2:** Participants’ physiological responses before and after walking on a treadmill in thermoneutral and warm conditions.

Variable	Thermoneutral condition		Warm air condition	
	Mean ± SD		Mean ± SD	
	Baseline	After activity	Baseline	After activity
Heart rate (bpm)	70 ± 13.16	113.30 ± 13.20	65 ± 15.20	122.15 ± 15.27
Skin temperature (°C)	33.68 ± 1.53	33.87 ± 1.55	35.12 ± 0.89	35.84 ± 0.89
Ear temperature (°C)	34.98 ± 0.56	35.40±0.60	35.64 ± 0.27	36.81 ± 0.29

Table 3 presented the pre-post change in body physiological responses before and after walking on a treadmill in thermoneutral and warm conditions. It can be seen that the HR and ST of the participants exposed to the warm air-condition increased by an average of 14 bpm and 0.75°C, respectively.

**Table 3:** The physiological response pre-post change before and after walking on a treadmill in thermoneutral and warm conditions.

Variable	Thermoneutral condition	Warm air condition	p-value
	Mean ± SD	Mean ± SD	
Heart rate (bpm)	43.3±13.20	57.15±15.27	<0.01
Ear temperature (°C)	0.42±0.2	1.17±0.33	<0.01

Figs 3 and 4 illustrated the significant correlation between one of the primary individual risk factors, VO_2_ max, and some important physiological responses (HR and ET) in a warm air condition. The Pearson test showed that the ET difference before and after walking on a treadmill was significantly correlated with VO_2_ max (r = -0.57, p<0.05). There was also a significant correlation between VO_2_ max and HR difference in the warm air condition (r = -0.59, p<0.05).

**Fig 3:** The scatter plots of theVO_2_ max compared to heart rate difference before and after walking on a treadmill in the warm air condition.

**Fig 4:** The scatter plots of the VO_2_ max compared to the ear temperature difference before and after walking on a treadmill in the warm air condition.

Pearson’s test showed that VO_2_max was significantly negatively correlated with the urinary density of participants in the warm air condition(r = -0.55, p<0.05). Fig 5 showed the correlation between VO_2_ max and urine-specific gravity of participants in warm air condition.

**Fig 5:** The scatter plots of the VO_2_ max compared to urine-specific gravity in the warm air condition.

### 3.2 Results of the LMM model

Table 4 presented the results of the developed linear mixed-effects model for the analysis of heat tolerance indicators. The model showed the effect sizes of main individual characteristics and thermal air condition on heat tolerance indicators. The developed model’s main input variables include BMI (in two levels of normal and abnormal), air temperature (in two levels of thermoneutral and warm air conditions), VO2 max, and body fat mass. The main output variables of the developed model are the primary heat tolerance indicators as HR and ET. The thermal air condition had the most significant effect on heat tolerance indicators, including HR and ET. The workers’ VO2 max and body fat mass was also identified as the main influential individual factors in HR. BMI had no significant effect on the body’s physiological responses of workers exposed to the thermal condition.

**Table 4:** The LMM model for analyzing the effects of body characteristics on heat tolerance indicators.

			Heart rate		Ear temperature	
			Estimate ± SE	p-value	Estimate ± SE	p-value
**Fixed Effects**	Predictors	Description				
	Intercept		187.39**±**18.03	<0.001	38.49**±**0.96	
	Air temperature	Warm (35°C)	9.11±1.58	**<0.001**	1.36±0.10	**<0.001**
		Thermoneutral (22°C)	Reference	--	Reference	--
	BMI	Abnormal (<18.5, >24.9)	-0.42±4.34	0.92	-0.06±0.22	0.79
		Normal (18.5 to 24.9)	Reference	--	Reference	--
	Vo_2_ max	(l/min)	-23.58±5.29	**<0.001**	-0.22±0.27	0.43
	Body fat mass	Kg	1.25±0.32	**<0.001**	0.00±0.01	0.64
**Random Effects**						
		Variance (SD)			Variance (SD)	
	Subjcts (Intercept)	58.83 (7.67)			0.144 (0.379)	
	Residual	26.46 (5.14)			0.112 (0.335)	
	Marginal R^2^ (Nakagawa)	0.63			0.685	

Figs 6 and 7 showed the measured values compared to the predicted values based on LMM for ET and HR. Based on the marginal(Nakagawa), the results confirmed the good performance of the developed LMM for predicting body heat tolerance indicators(R^2^ = 0.63 and 0.685).

**Fig 6:** The ear temperature (ET) measured values compared to the predicted values based on LMM.

**Fig 7:** The heart rate (HR) measured values compared to the predicted values based on LMM.

## 4 Discussion

The current study investigated the effect of different influential risk factors on the body heat tolerance of workers exposed to a simulated warm working environment. Our results demonstrated that the heat tolerance indicators, including HR, ET, and ST, increased significantly in the warm air condition compared to the thermoneutral condition. According to the results of the LMM model, the air temperature had the most significant effect on body physiological responses, including HR and ET. It is noteworthy that considering the same workload (moderate working metabolism) in both thermoneutral and warm conditions, the HR of subjects exposed to warm air conditions increased by an average of 14 bpm. As a result, participants experienced light cardiovascular strain, which should be considered by occupational hygienists to monitor the health of workers exposed to heat in typical light metal industries and similar industries.

Moreover, the ET of participants exposed to warm air conditions increased by an average of 0.75°C. According to ISO 9886, the limit value of the physiological thermal strain for workers was determined body temperature increase by about one degree Celsius in less than one hour. In the present study, during the 30 min exposure of workers to heat, their body temperature increased by an average of 0.75°C, that this important finding should be considered by occupational hygienists and managers that determine the permissible limits of exposure to heat. These findings of the effects of exposure to warm air conditions on HR and ET are consistent with some studies’ results [16, 26, 46–48]. It should be noted that the use of ET as a relatively reliable indicator of thermal strain is recommended by the United Kingdom Institute for Occupational Medicine for the Health and Safety Executive in accordance with the standard measurement method [49].

As displayed in Table 4, after ambient air temperature, VO_2_ max had a significant effect on the HR of the participants. As presented in Fig 3, participants with a higher VO_2_ max had a slower HR when exposed to warm air condition. Lisman et al. indicated that VO_2_ max was also the most influential factor in HR and core body temperature during the heat tolerance test [26]. According to the results of the LMM model (Table 4), VO_2_ max did not significantly affect ET. Nonetheless, as demonstrated by Fig 4, the difference in ET before and after walking on a treadmill in the warm air condition was significantly negatively correlated with VO_2_ max. In other words, participants with higher aerobic capacity had lower body temperatures. Coso et al. reported that heat dissipation exceeds heat accumulation in people with higher aerobic capacity engaged in exercises with the same intensity [50]. Lu et al. demonstrated that the VO_2_ max was influential in the physiological response to the warm air condition [16]. It seems that the considered exposure time (30 minutes) is not enough to make some remarkable ear temperature responses in the warm air condition compared with the heart rate responses. Due to the possibility of missing the participants in longer exposures, 30 minutes of exposure was considered in each experimental session. Moreover, it can be seen that the heart rate might be a generally more sensitive indicator than body temperature to incremental changes in air temperature.

According to the results of the LMM model, body fat mass significantly affected the HR of the participants. In this regard, participants with a higher body fat mass had a higher HR. In agreement with our findings, Dehghan et al. reported that the intensity of heat strain was higher in overweight workers [51]. Lu et al. also reported that body surface area and fat percentage were influential in the physiological response to heat [16].

The measuring of physiological responses in the warm air condition showed that none of the physiological responses significantly differed based on BMI. However, descriptive results indicated that participants with normal BMI have a higher aerobic capacity, lower fat percentage, and higher heat tolerance than those with abnormal BMI. Most participants in the present study had normal BMI, so there was no significant difference in physiological responses based on BMI. It is proposed that a broader variation in BMI distribution for a more comprehensive study.

It is observed that there was no significant difference between urinary density in thermoneutral and warm conditions (Table 2). However, as shown in Fig 5, participants with higher aerobic capacity had lower urine density in the warm air condition. Since urine density is considered an indicator of hydration status [42], participants with higher aerobic capacity had better hydration. Batista et al. demonstrated that hydration was influential in the aerobic capacity of athletes [52]. It should be noted that urine-specific gravity is widely accepted as a convenient and reliable indicator of hydration status. However, two thermal air conditions considered in this study cannot affect participant hydration status significantly.

The current finding showed that the developed linear mixed model accurately estimates body heat tolerance with different influential risk factors. It can be a helpful screening tool for properly selecting workers in occupational medical examinations for working in warm air conditions. However, the domain of this analysis model is restricted to a defined air temperature range. The air temperature range was selected based on thermal air conditions of the typical real warm metal industry. However, some physiological responses did not show considerable variations in this climatic condition. This model can be expanded for warmer to hot air conditions of the typical working environment.

Future studies can also investigate the effect of the aerobic capacity of workers on other sensitive physiological responses such as heart rate variability, urine osmolality, and sweat characteristics in similar thermal condition of the current study. The present study was based on short-term exposure to thermal conditions while working hours are longer in the real world. The possibility of conducting a field study under controlled other environmental conditions is limited. Hence, field studies with long-term exposure to the same thermal conditions are recommended to verify these findings.

## 5 Conclusions

The analysis model for body heat tolerance verified that individual characteristics of workers as aerobic and physical fitness, have a critical role in reducing physiological strain in warm environments. Improving the workers’ aerobic capacity through regular exercise programs and lifestyle modifications can strengthen body heat tolerance. The selection of workers with good aerobic fitness during an occupational medical examination for working in warm air conditions will mitigate the risk of heat-related illness.

## Supporting information

S1 Data (XLSX)
